# Significance of Continuous Nursing of Omaha System in Children after Hypospadias Surgery and Its Influence on Infection Complications

**DOI:** 10.1155/2022/8346848

**Published:** 2022-09-01

**Authors:** Junting Li, Xiaochen Fan, Qifei Deng, Jingjing Sun, Liping Jin, Peipei Chen, Pinglian Wei, Annuo Liu

**Affiliations:** ^1^Nursing School of Anhui Medical University, Hefei, Anhui 230061, China; ^2^Pediatric Urology Surgery, Anhui Provincial Children's Hospital, Children's Hospital of Fudan University-Anhui Campus, Hefei, Anhui 230051, China; ^3^Pediatric Intensive Care Unit, Anhui Provincial Children's Hospital, Children's Hospital of Fudan University-Anhui Campus, Hefei, Anhui 230051, China; ^4^Cardiovascular Department, Anhui Provincial Children's Hospital, Children's Hospital of Fudan University-Anhui Campus, Hefei, Anhui 230051, China; ^5^Comprehensive Pediatric Ward, Anhui Provincial Children's Hospital, Children's Hospital of Fudan University-Anhui Campus, Hefei, Anhui 230051, China

## Abstract

**Objective:**

The aim of the research article is to explore the significance of continuous nursing of the Omaha system in children after hypospadias surgery and its influence on infection complications.

**Methods:**

From April 2019 to April 2021, Anhui Provincial Children's Hospital treated 76 children with hypospadias and they were selected as the research objects. In the light of the random number table method, children were classified into the control group and the study group, with 38 cases in each group. The control group applied routine postoperative nursing intervention, while the study group received Omaha system continuous nursing intervention based on the control group. The Omaha system outcome evaluation, complication rate, quality of life, and nursing satisfaction were recorded and discussed in all children.

**Results:**

The levels of physiological and psychological environment and health behavior in both groups after intervention were significantly higher than those before the intervention, and the levels of all dimensions in the study group were significantly higher than those in the control group (*P* < 0.05); the complication rate in the study group was 10.53% significantly lower than that in the control group (28.95%). After intervention, the physiological function, psychological and social function, emotional function, social interaction, and school status of the two groups were significantly higher than before intervention, and the score of each dimension in the study group was significantly higher than that in the control group (*P* < 0.05); the overall satisfaction of nursing in the study group was 94.74% significantly better than in the control group (81.59%) (*P* < 0.05).

**Conclusion:**

The continuous nursing intervention of the Omaha system for children with hypospadias can significantly improve the clinical condition of children, reduce the risk of infection complications, improve children's physical and mental health status, and improve nursing satisfaction, which is worthy of clinical practice.

## 1. Introduction

Hypospadias is a congenital defect of male urinary system abnormalities, mainly occurring in children at the opening below the urethra and penis, manifested as ectopic urethra opening, abnormal curvature of the penis, abnormal prepuce, etc. In severe cases, indirect inguinal hernia will be induced. This disease belongs to external genital defect disease and is hereditary. When pregnant women have a family genetic history or are sick during pregnancy, neonatal hypospadias will significantly increase, affecting the healthy development of children, etc. [1, 2]. Clinical treatment for children with hypospadias is mainly surgical, including penile curvature correction, urethral molding, etc. In view of the rapid growth and development of children, long-term sustained and phased treatment is generally adopted to ensure the functional integrity of males in the future [3]. Relevant studies have shown [4] that after hypospadias in children, complications such as abnormal urination, urinary tract infection, and urethral stricture will be caused due to residual penis curvature and dry occlusive penile head infection. Postoperative complications of hypospadias will seriously affect the urination function, future sexual function, and mental health of children. In addition, due to the immature mind and young age, poor compliance during treatment significantly increases the difficulty of postoperative nursing, which is not conducive to the prognosis and rehabilitation effect. Therefore, it is necessary to take scientific and reasonable postoperative care for children undergoing hypospadias [5, 6].

Routine clinical nursing only ensures the risk of complications in children during treatment, observes the short-term development direction of the disease, and has no observation index for functional testing of adult males [7]. As a clinical nursing model approved by the American Nursing Association, the Omaha system can analyze and sort out problems during nursing and implement the personalized, systematic nursing intervention. Reasonable evaluation of nursing intervention results has been widely used in nursing research and obtained significant application value. However, there is still limited literature on continuous nursing of hypospadias in clinical practice, and no specific research indexes and other research projects have been found [8, 9]. Based on the research status at home and abroad, this study implemented the Omaha system of continuous nursing intervention for children undergoing hypospadias, aiming to observe Omaha outcome evaluation, complications, quality of life, and nursing satisfaction, and the report is as follows.

## 2. Data and Methods

### 2.1. General Information

  From April 2019 to April 2021, seventy-six children treated at Anhui Provincial Children's Hospital undergoing hypospadias were selected as the study objects. Patients were divided into control group and study group based on length of hospital stay, all of whom were male. The control group was 2.26–4.05 years old, with an average age of (3.21 ± 0.61) years, and the course of illness was (2.42 ± 0.59) months. The age of the study group ranged from 2.31 to 4.03 years, with an average (3.19 ± 0.59) years and the course of disease of (2.40 ± 0.58) months. Clinical data on both, including gender and age, and other general data were not significantly different (*P* > 0.05). The control group took routine postoperative nursing intervention, and the study group took Omaha system of continuous nursing intervention on the basis of the control group. The hospital's medical ethics committee approved our study.

### 2.2. Inclusion and Exclusion Criteria

Inclusion criteria were as follows: ① comply with Practical Pediatric Urology about the standard of diagnosis of hypospadias [10]; ② congenital hypospadias was confirmed by physical examination, genital ultrasound, and chromosome examination; ③ the first transurethral hypospadias surgery; ④ age ≤12 years; ⑤ complete clinical data; ⑥ the family members of children with no cognitive impairment and mental disorders. The children and their statutory guardian were informed of the research contents and provided informed consent forms.

Exclusion criteria were as follows: ① patients with hematological system and autoimmune system disorders; ② patients with serious dysfunction of the heart, liver, and lung; ③ complicated with urethral stricture, urethral diverticulum, and other diseases; ④ contraindications associated with surgery; (5) history of urethral surgery; ⑥ the patient's family members cannot follow the doctor's advice and do not cooperate with the follow-up schedule.

### 2.3. Research Methods

The control group was given routine nursing care, including physical examination, reproductive organ ultrasound, and chromosome examination, during hospitalization. During hospitalisation, the control group received regular nursing care such as physical examination, reproductive organ ultrasonography, and chromosomal examination. supervise children's daily diet, physical activity, drug control, and nursing guidance, as well as dynamic monitoring of clinical indicators such as temperature, skin status, blood pressure, and electrocardiogram. Health education, medication instructions, and nursing guidance were given to the family members and caregivers before discharge. Before discharge, family members and caregivers are given health education, medication instructions, and nursing assistance. Monthly regular review or follow-up after discharge, children's test-related indicators, informing the disease control situation and the next nursing plan, abnormal conditions during discharge, going to the hospital on time, and frequent review once the condition are stable. The study group adopted the Omaha system of continuous nursing intervention based on routine nursing care. The concrete contents are as follows: (1) The Omaha system continuity care team was established, with members including 1 attending doctor, 2 chief nurses, 6 experienced nursing staff, 1 child dietitian, 1 psychological consultant, and 1 rehabilitation consultant. The nursing team members were organized to learn the intervention significance, concept, project-specific content, implementation process, and successful cases of Omaha system continuity care, and they were asked to enter the job after passing the assessment. Responsibilities of group members: as the head of the group, the chief nurse and the attending doctor will coordinate the overall nursing progress, timely improve the nursing plan according to specific feedback, and be responsible for the study, investigation, and review of group members. The nursing staff consulted the data, combined the situation of children in the hospital and their personal experience, summarized the causes, mechanisms, common solutions, and efficacy of complications in children undergoing hypospadias, implemented specific nursing programs, and provided timely feedback, summary, and analysis. (2) Specific operation process: ① Problem summary: According to access to data, clinical data summary, and the use of Omaha system problem classification, potential nursing problems are summarized, including psychosocial, physiological, behavioral, and environmental four aspects, according to the theory of demand to develop nursing priorities. In addition, based on the clinical symptoms and physiological needs of the children, personalized problems were screened out, including nutritional status, psychological status, and physical signs, and the nursing problems and nursing direction of the children were summarized. ② Intervention measures: children and their relatives' information files, according to the children's age, height, weight, symptoms, eating habits, and other targeted nursing interventions, control children's medication, diet, exercise, and psychological and social state and record the nursing process and nursing effect. During hospitalization, the nursing staff communicated with the children as much as possible. With the help of toys, picture books, etc., children can increase their sense of familiarity and intimacy with wards and doctors. Through different games to increase children's understanding of the disease, reduce their resistance, and improve their psychological disorders and bad emotions, the nurses could increase their cooperation and enthusiasm for nursing projects, give positive health publicity and nursing guidance to children's relatives, correct their bad parenting views and nursing measures, and relieve their depression, anxiety, and other negative emotions; After discharge, an Internet platform system group chat was established to increase the contact between relatives of children. They were asked to encourage each other and share experiences to create a positive nursing atmosphere. To push internet groups on a regular basis on health care knowledge, precautions, such as recording, guiding families with medication, exercise, and diet, improving children's ability with self-initiative and management, if haemorrhage, infection, and so on can be reserved for pharmacist calls or Internet communication platforms after hospital doctors discuss appropriate antibiotics to control, reduce their anxiety, and enhance nurse compliance. ③ Effect evaluation: follow-up by telephone or SMS or outpatient visit can be done after the implementation of specific measures, and the follow-up time is arranged as a weekly follow-up. The duration lasted for 4 weeks, and the nursing adaptation, physiological status, and disease control were mainly observed. After that, the patients were followed up every two weeks for 8 weeks, mainly observing psychological and physical status and social relationships. After that, the patients were followed up once a month for three months to observe the role problems with family and society, psychological adaptability, and nursing effect. During the follow-up period, the Omaha outcome scoring system was used to evaluate the nursing effect, and the nursing plan and measures were adjusted for renursing intervention if the effect was not good.

### 2.4. Observation Indicators

① Omaha system score: The effect of the intervention was evaluated by the Omaha system, and Likert's 1 ∼ 5 rating method evaluated the cognition, behavior, and children's living status. The results were divided into four dimensions, including physiological, psychological, environmental, and health behavior. The lower the score is, the less significant the disease intervention effect is and the scoring system is more authoritative and feasible. ② Complication rate: after a follow-up period of 6 months, our study recorded complications, including infection, redness and bleeding, urinary fistula, urethral diverticulum, and urethral stricture. ③ Comparison of living quality: the Pediatric Quality of Life Inventory (PedsQL) [11] was applied to evaluate patients' living quality in the two groups before intervention and 6 months after intervention. The scale was evaluated by parents and children, respectively, with a total of 5 aspects, including physiological function, psychological and social function, emotional function, social interaction, and school state. There are 23 items on a scale of 0 to 100; the higher the score, the better the quality of life. The internal consistency reliability of the scale is 0.789, which is an effective and reliable measurement tool. ④ Overall nursing satisfaction: according to the nursing resources and level of our hospital and the Nursing satisfaction Questionnaire of Newcastle (NSNS) [12], we prepared a Nursing Satisfaction Scale with a total of 20 questions. A five-level scoring method was adopted, and the total score was 20–100, of which 90–100 was very satisfied, 75–89 was relatively satisfied, 60–74 was satisfied, and 20–59 was dissatisfied. Overall satisfaction = (very satisfied + relatively satisfied + satisfied) cases/total cases × 100%.

### 2.5. Statistical Treatment

SPSS 24.0 statistical software was applied. Measurement data were expressed as $\bar{x}\pm s$, count data were expressed as a percentage, and statistical analysis was performed by *t*-test, *Z* test, and *χ*^2^ test. *P* < 0.05 was considered statistically significant.

## 3. Results

### 3.1. Comparison of Basic Data between the Two Groups

The results showed that gender, age, course of the disease, disease type, hypocleft type, birth mode, guardian education level, and other basic information were compared between the two groups. The difference was not statistically significant (*P* > 0.05), as shown in Table 1.

### 3.2. Comparison of Omaha System Scores between the Two Groups

Results showed that the Omaha system score between the two groups showed no significant difference before intervention (*P* > 0.05). The levels of physiological and psychological environment and health behavior in both groups after intervention were significantly higher than those before intervention, and the levels of all dimensions in the study group were significantly higher than those in the control group (*P* < 0.05), as shown in Table 2.

### 3.3. Comparison of Complication Rates between the Two Groups

The results showed that the complication rate in the study group was 10.53% significantly lower than that in the control group (28.95%). The difference was statistically significant (*P* < 0.05), as shown in Table 3.

### 3.4. Comparison of Quality of Life between the Two Groups

The results showed that there was no significant difference in quality of life between the two groups before intervention (*P* > 0.05). After intervention, the physiological function, psychological and social function, emotional function, social interaction, and school status of the two groups were significantly higher than before intervention, and the score of each dimension in the study group was significantly higher than that in the control group, as shown in Table 4.

### 3.5. Comparison of Total Nursing Satisfaction between the Two Groups

Results suggested that the overall satisfaction of nursing in the study group was 94.74% significantly better than in the control group (81.59%) (*P* < 0.05), as shown in Table 5.

## 4. Discussion

Hypospadias is one of the common diseases in pediatric urology, which is mostly related to heredity, gene mutation, and pregnancy status. No studies have clearly explained its pathogenesis and mechanism. According to epidemiological data [13], the incidence of neonatal hypospadias accounts for the second place among birth defect diseases, with a domestic incidence of 0.91%, which seriously affects the urinary function of children and adult males. Operation is the main treatment for children with hypospadias, and there are many clinical treatment methods. However, due to the unique physiological structure and limitations of children, postoperative infection complications are prone to occur, which seriously affects the treatment effect and overall treatment rate [14–16]. Therefore, the prevention and treatment of complications in children with hypospadias can significantly reduce the clinical symptoms and adverse reactions and improve the prognosis. The Omaha system of continuous care will be problem classification, intervention measures, and effect detection as a subsystem-combined application, to establish a complete, scientific, operational strong nursing system, which has been widely used in education, scientific research, and other fields. Relevant studies have shown [17] that the system has developed a systematic operation process in the prevention and care of complications of chronic diseases such as diabetes and stroke, which has considerable scientific research prospects. The purpose of this study was to apply the Omaha system of continuous care to children undergoing hypospadias and effectively improve their quality of life. And to control the prognosis effect, lower the incidence of postoperative morbidity, and meet the needs of children and their families for nursing work, nursing effect is significant.

The postoperative complications of hypospadias, such as infection, redness, and bleeding, are easily disturbed by the anatomical structure and psychological tolerance of children. In addition, inadequate postdischarge nursing measures and limited cognition of family members will also cause long-term complications, such as urinary fistula and urethral stricture, which will have serious adverse effects on the physiology and psychology of children [18]. Peng L et al. [19] used the Omaha system for nursing management of chronic kidney disease patients undergoing peritoneal dialysis. It can obviously control the nutritional status of patients, maintain physical health and improve quality, reduce the risk of cardiovascular complications, control mortality and morbidity, and achieve better nursing effects; Liu et al. [20] applied the Omaha system of continuous care to intervene in patients with double-J tube retention after urinary calculus surgery, which can relieve patients' depression, worry, and other negative induced moods and perfect their sleep quality and life quality. In the study, the levels of physiological and psychological environment and health behavior in both groups were significantly increased after intervention; compared with the control group, the levels of all dimensions in the study group were significantly higher, and the complication rate of the study group was significantly lower. This is consistent with the results of Peng and Liu et al. This indicates that the Omaha system of continuous care for children undergoing hypospadias can significantly improve nursing efficiency and reduce the incidence of infection complications. The Omaha system combines problem classification, intervention, and outcome assessment to predict adverse events and complications that may occur during care. According to the relevant psychological guidance, intervention measures improve the children's trust in the nursing staff and work and increase the compliance during nursing. In addition, through supervision of children's reasonable diet, exercise, and medication control, it can improve the level of self-management during the nursing of children, promote the smooth development of continuous care in the Omaha system, improve the health status of children, and effectively control the risk of infection complications from the source.

The living quality scale was applied widely to clinical study and can significantly assess the pain degree and functional level of children, practice, and community investigation with high reliability and validity [21]. ording to Zhuang et al. [22], the Omaha system of continuous care may enhance the psychological status, self-esteem, and quality of life of children with epilepsy, resulting in ideal intervention effects.Acc The results showed that after intervention, the physiological function, psychological and social function, emotional function, social interaction, and school status of both groups were significantly better than before intervention and the study group's score was significantly higher than that of the control group. Compared with the control group, overall nursing satisfaction of the study group was significantly higher. The results are similar to the study by Zhuang et al., showing that the Omaha system can significantly improve the quality of life of children after hypospadias and improve the overall care satisfaction of children and their families. Omaha's system of continuous care by regularly explaining the concept of disease, nursing measures, and precautions to children and their relatives, urging timely medication, exercise, etc. through long-term intervention to regulate children's physical condition and disease cognition; improve children's mental health; boost their sense of self-worth; alleviate negative emotions; promote physical, psychological, social relationship, and learning state; and increase nursing satisfaction. In addition, Omaha nursing adopts stage effect evaluation and timely adjustment of the nursing program to meet the needs of children and their families for nursing services, achieve sustainable nursing program, decrease the risk of postoperative complications, and improve their quality of life and nursing recognition [23].

In conclusion, the Omaha system's continuous nursing intervention after hypospadias in children can effectively improve their disease cognition and nursing recognition, improve their physical, psychological, and social roles and health behaviors, and reduce the incidence of infection complications. Furthermore, providing a reference increases the quality of life and overall nursing satisfaction for clinical hypospadias postoperative nursing. However, expanding the sample size to further explore the universal adaptability and feasibility of this nursing model is quite necessary. In addition, there is no accurate operation process and standard in this study, so we need to consult the data and clinical research to find out the standard process and indicator standard.

## Figures and Tables

**Table 1:** Comparison of baseline data of two groups of children.

Group		Control group (*n* = 38)	Study group (*n* = 38)	Statistics	*P*
Gender (case, *n*, %)	Male	38(100.00)	38(100.00)	2.162	0.064
	Female	0(0.00)	0(0.00)		

Average age (years, $\bar{x}\pm s$)		3.21 ± 0.61	3.19 ± 0.59	0.192	0.109

Mean course of disease (months, $\bar{x}\pm s$))		2.42 ± 0.59	2.40 ± 0.58	0.427	0.071

Disease types (case, *n*, %)	Penis head type	18(47.37)	17(44.74)	0.418	0.115
	Penis size	16(42.11)	15(39.47)		
	Penile scrotal type	3(7.89)	5(13.16)		
	Perineum type	1(2.63)	1(2.63)		

The split type (case, *n*, %)	I	12(31.58)	11(28.95)	0.439	0.058
	II	18(47.37)	20(52.63)		
	III	5(13.16)	5(13.16)		
	IV	3(7.89)	2(5.26)		

Born way (case, *n*, %)	Natural birth	21(55.26)	23(60.53)	0.637	0.136
	Caesarean section	17(44.74)	15(39.47)		

Guardian educational level (example, *n*, %)	High school and below	5(13.16)	7(18.42)	0.116	0.072
	Undergraduate and junior college	19(50.00)	18(47.37)		
	Postgraduate and above	14(36.84)	13(34.21)		

**Table 2:** The comparison of Omaha system score between the two groups ($\bar{x}\pm s$, points).

Group	Time	Control group (*n* = 38)	Study group (*n* = 38)
Physiological	Before the intervention	8.32 ± 2.07	8.32 ± 2.13
	After the intervention	9.17 ± 2.11^*∗*^	12.95 ± 2.16^*∗*#^

Psychological	Before the intervention	8.06 ± 2.02	8.06 ± 2.01
	After the intervention	9.23 ± 2.15^*∗*^	11.63 ± 2.13^*∗*#^

Environment	Before the intervention	7.94 ± 2.10	7.93 ± 2.08
	After the intervention	9.54 ± 2.16^*∗*^	13.57 ± 2.21^*∗*#^

Health behavior	Before the intervention	8.13 ± 1.93	8.14 ± 1.96
	After the intervention	9.83 ± 1.98^*∗*^	11.42 ± 2.02^*∗*#^

*Note.* Compared with before intervention, ^*∗*^*P* < 0.05. Compared with the control group before intervention, ^*∗*#^*P* < 0.05.

**Table 3:** Comparison of complication rates (cases, %).

Group	Control group (*n* = 38)	Study group (*n* = 38)	*χ* ^2^	*P*
Infection	3(7.89)	1(2.63)	—	—
Red bleeding	4(10.53)	2(5.26)	—	—
Urinary fistula	1(2.63)	0(0.00)	—	—
Urethral diverticulum	1(2.63)	1(2.63)	—	—
Urethral stricture	2(5.26)	0(0.00)	—	—
Complication rate	28.95%	10.53%	2.310	0.015

**Table 4:** Comparison of quality of life level ($\bar{x}\pm s$, points).

Group	Time	Control group (*n* = 38)	Study group (*n* = 38)
Physiological function	Before the intervention	43.26 ± 10.69	43.30 ± 10.67
	After the intervention	51.09 ± 12.04^*∗*^	56.93 ± 13.28^*∗*#^

Psychological and social function	Before the intervention	45.62 ± 11.07	45.68 ± 11.21
	After the intervention	49.86 ± 12.52^*∗*^	55.94 ± 14.47^*∗*#^

Emotional function	Before the intervention	59.66 ± 13.62	59.27 ± 13.45
	After the intervention	65.32 ± 15.18^*∗*^	78.72 ± 17.62^*∗*#^

Social interaction	Before the intervention	47.62 ± 11.36	47.75 ± 11.41
	After the intervention	56.38 ± 13.94^*∗*^	68.95 ± 15.71^*∗*#^

State of the school	Before the intervention	49.63 ± 10.15	49.85 ± 10.27
	After the intervention	54.87 ± 12.26^*∗*^	66.43 ± 14.58^*∗*#^

*Note.* Compared with the control group before intervention, ^*∗*#^*P* < 0.05.

**Table 5:** Comparison of total nursing satisfaction (example, %).

Group	Control group (*n* = 38)	Study group (*n* = 38)	*χ* ^2^	*P*
Very satisfied	16(42.11)	19(50.00)	—	—
Generally satisfied	9(23.68)	11(28.95)	—	—
Satisfied	6(15.79)	6(15.79)	—	—
Not satisfied	7(18.42)	2(5.26)	—	—
Complication rate	81.59%	94.74%	0.391	0.007

## Data Availability

The data used to support the findings of this study are available from the corresponding author upon request.
